# The Differences in Clinical Characteristic and Outcomes of New Onset Typical versus Atypical Right Branch Bundle Block in Acute Myocardial Infarction

**DOI:** 10.1155/2022/4620881

**Published:** 2022-08-31

**Authors:** Jingchao Li, Luqian Cui, Lingkun Ma, Haijia Yu, Huihui Song, Shujuan Dong, Yingjie Chu

**Affiliations:** ^1^Department of Cardiology, Henan Provincial People's Hospital, Zhengzhou, Henan 450003, China; ^2^Department of Emergency, Henan Provincial People's Hospital, Zhengzhou, Henan 450003, China

## Abstract

**Objective:**

The purpose of this study is to explore the clinical characteristics and estimate the new-onset atypical right branch bundle block (ATRBBB) predictive value in short-term and long-term mortality by comparing the typical right branch bundle block (TRBBB) subset in acute myocardial infarction (AMI) patients.

**Methods:**

A total of 224 AMI patients combined with new onset RBBB who received primary coronary angiography were included, being admitted to Henan Provincial People's Hospital in China from July 2010 to June 2021. Patients were divided into typical RBBB group (*n* = 104) and atypical RBBB group (*n* = 120). The differences in clinical characteristics between the two groups were analyzed. Logistic and Cox regression analysis were performed to identify independent predictors of in-hospital Major Adverse Cardiovascular Events (MACE).

**Result:**

The ATRBBB group had a higher proportion of smoking and alcohol consumption, higher body mass index, worse cardiac function (killip ≧ II proportion), higher peak value of CK-MB, lower LVEF%, longer total ischemia time, higher proportion of LAD (left anterior descending coronary artery) occlusion, and multivessel lesions, compared to the TRBBB group. The ATRBBB group had a higher proportion of in-hospital MACE and 1-year all-cause mortality compared to the TRBBB group. ATRBBB was an independent predictor of in-hospital MACE and 1-year mortality in patients with AMI combined with new onset RBBB.

**Conclusions:**

ATRBBB group had more serious clinical symptoms and clinical prognosis. New ATRBBB is an independent predictor of in-hospital MACE and 1-year death in patients with AMI combined with RBBB. If the infarct-related vessel was opened immediately, the evolution of TRBBB to ATRBBB may be avoided, leading to a better prognosis.

## 1. Introduction

Acute myocardial infarction (AMI) is the most severe cardiovascular disease threatening human health, characterized by rapid onset, fast development, and high mortality [1]. With the popularization of primary coronary interventional (PCI) therapy, the survival rate of AMI has been greatly improved [2]. Nevertheless, AMI combined with branch bundle block (BBB) still has a high mortality rate as a special population [3]. Although numerous studies have proposed that AMI combined with BBB patients has a poor prognosis [4, 5], previous AMI guidelines only mentioned new-onset LBBB as the indication for the early diagnosis of AMI and emergency revascularization [6, 7]. 2017 ESC STEMI guidelines listed new-onset RBBB as an indication for emergency revascularization. From then on, mainstream guidelines have been updated successively [8]. Changes in guidelines indicate the important values of new-onset RBBB in the diagnosis and treatment of AMI.

Our research team has been paying attention to the value of newly emerging RBBB in the early diagnosis of AMI for many years [9]. According to our clinical observation and follow-up, we found that the ECG characteristics of AMI combined with RBBB were different. Some patients present qRBBB, including q/Q waves in the right precordial or anterior septum leads (we named it atypical RBBB); the other patients present rsR (we name it typical RBBB) and there may exist differences in basic clinical characteristics, coronary artery lesions, and clinical prognosis.

Although previous studies suggested that AMI combined with RBBB has poor prognostic [10], especially qRBBB [11], no literature has been published focusing exclusively on a different type of RBBB and given a clear definition of AMI with typical RBBB (TRBBB) and atypical RBBB (ATRBBB) in the ECG. Therefore, we conducted a retrospective study of all patients who presented with AMI combined with new-onset RBBB, dividing them into typical RBBB group and atypical RBBB group according to the different forms in the ECG, focusing on the difference in their basic clinical characteristic, ECG, angiographic profile, the in-hospital MACE, and 1-year mortality. The main objectives of the study were to distinguish the clinical characteristics and estimate the new-onset ATRBBB predictive value in short-term and long-term mortality by comparing the TRBBB subset in AMI patients.

## 2. Materials and Methods

### 2.1. Study Design and Patients

This was a single-centre retrospective study; a total of 2813 consecutive patients with AMI [12, 13] who received emergency PCI routinely admitted to Henan Provincial People's Hospital in China from July 2010 to June 2021 were retrospectively collected, 273 patients combined with RBBB in the ECG, 237 patients' RBBB in the ECG was new onset, and only 224 patients who combined with new onset RBBB having integral material entered the final analysis. Patients were divided into TRBBB group and ATRBBB group according to the ECG characteristics.

Inclusion criteria were as follows: (1) Patients were aged ≥18 years. (2) Patients were diagnosed as AMI combined with new onset RBBB. If the patient can provide normal ECG without RBBB within six months or confirm not having medical history of RBBB, we define the ECG with RBBB as new onset. (3) Patients were admitted within 24 hours to the Emergency department. Exclusion criteria were as follows: (1) patients who were documented to have preexisting RBBB before the hospital admission; (2) the IRA being LM; (3) patient with severe liver and kidney dysfunction, advanced malignant tumor, and active bleeding; (4) patient with a life expectancy <1 year; (5) patients with any pattern of BBB other than RBBB pattern.

Baseline data such as age, gender, body mass index (BMI), unhealthy habits (smoking, alcohol), comorbidities (hypertension, diabetes, hyperlipemia), preoperative cardiac function grade (Killip ≧ II), peak value of creatine kinase isoenzyme (CK-MB), left ventricular ejection fraction (LVEF), and total ischemia time (TIT) of all included patients were recorded. The study was approved by the institutional review board and the ethics committee of Henan Provincial People's Hospital (2020-158).

### 2.2. Classification Standard of ECG

Patients were divided into TRBBB group and ATRBBB group according to the ECG characteristics. TRBBB diagnostic criteria were as follows: (1) QRS group time ≥120 ms. (2) The wave form of QRS in lead *V*_1_ or *V*_2_ is rsR′ type or M type, which is the most characteristic change (Figure 1(a)); the lead S waves of I, V_5_ and V_6_, are broadened with notch, and the time limit is ≥40 ms; the avR lead is of QR type, and its R wave is broadened and truncated. (3) V_1_ lead R peak time ≥50 ms. (4) ST segment of V_1_ and V_2_ leads was slightly depressed, with negative T wave; and the direstion of T wave in I, V5, and V6 leads was opposite to S wave, but still upright. ATRBBB diagnostic criteria were as follows: (1) QRS broadening ≥120 ms. (2) The QRS wave of V_1_ or V_2_ is qR′ or R type (Figure 1(b)). (3) It does not meet the diagnostic criteria of TRBBB. All patients received 12-lead ECG when they arrived in the emergency room in this study, and 18-lead ECG was added in patients with high suspicion of posterior and inferior MI. ECG records were obtained on admission, 10–20 minutes later, after reperfusion therapy, every 6 hours on day 1, twice daily on day 2, and daily thereafter until discharge. If the RBBB appeared after admission or was present on admission but was not recorded on an ECG performed within the previous 6 months, it was defined as new onset. New-onset RBBB was further classified as transient if it disappears when the patient is discharged and permanent if it still exists when the patient dies or is discharged.

### 2.3. Coronary Angiography and Intervention

The emergency coronary angiography (CAG) results of all patients were reviewed and recorded by 2 experienced interventional cardiologists, including the infarct-related vessels (IRA), the number of vascular lesions, IRA proximal occlusion or not, the proportion of IRA anterior TIMI flow 0/1, and whether emergency stents placement was performed.

### 2.4. Follow-Up and Outcome

Patients were followed up by a dedicated nursing team until the time of an event happened or, in the case of no event, 365 days. The follow-up method included having a telephone interview with the patients or with a close family member and/or having a review of the medical record. The primary endpoint was all-cause mortality during one-year follow-up. The second endpoint was the incidence rate of in-hospital MACE.

The incidence of in-hospital major adverse cardiac events (MACE) and 1-year mortality were recorded. In this study, MACE was defined as cardiogenic shock, malignant ventricular arrhythmias (ventricular tachycardia, flutter, and ventricular fibrillation), second-degree type II or above atrioventricular block (AVB), in-hospital recurrent AMI, cardiogenic stroke, and sudden cardiac death. The 1-year follow-up was conducted by telephone, and the endpoint of event was all-cause death.

### 2.5. Statistical Analysis

Statistical analysis of the acquired data was done using SPSS 23.0 software (SPSS Inc., Chicago, Illinois). Acquired data were summarized using mean with standard deviation (SD) or median with interquartile range. Continuous variables were compared using an independent Student's *t*-test for variables with normal distribution and Man-Whitney *U* tests for those with nonnormal distribution. The *χ*^2^ test was used for categorical variables. Logistic regression analysis was done to identify the independent predictors of in-hospital MACE of AMI patients with new-onset RBBB, and Cox regression analysis was done to identify independent predictors of 1-year mortality of AMI patients combined with new onset RBBB. Odds ratio (OR), hazard ratio (HR), and corresponding 95% confidence intervals (95% CI) are presented as effect estimates. *P* < 0.05 was considered to be statistically significant.

## 3. Results

### 3.1. Patients' Information

A total of 224 AMI patients with RBBB were included in this study: 104 patients in the TRBBB group and 120 patients in the ATRBBB group. Baseline clinical characteristics are presented in Table 1. The mean age was 66.2 ± 12.19 years, and 72.8% of patients were male, while 27.2% were female. The ATRBBB group patients have higher BMI, a higher ratio of alcohol and smoking, worse heart function (higher ratio of Killip level ≥ II), lower LVEF%, and longer TIT compared to the TRBBB group, and there were statistical differences (*P* > 0.05).

### 3.2. ECG Characteristic

In this study, the ECG characteristics of patients in the two groups were compared and the ECG characteristic differences are shown in Table 2. Dynamic monitoring of ECG of the two groups showed that the ATRBBB group had a higher proportion of anterior wall/anterior septum/extensive anterior wall myocardial infarction, and the difference between TRBBB and ATRBBB has a statistical value (*P* < 0.05). The TRBBB group had a higher proportion of transient new RBBB compared to the ATRBB group (*P* < 0.05), while there was no significant difference in the proportion of ST-segment elevation between the two groups (*P* < 0.05).

### 3.3. Coronary Angiography Characteristics and Percutaneous Coronary Intervention

The characteristics of coronary artery lesions were compared between the two groups, and the coronary artery lesions' characteristics are shown in Table 3. Coronary angiography results showed that occlusive conditions in both groups were mostly proximal to IRA, and the main coronary artery lesions in 214 AMI patients were left anterior descending (LAD) coronary artery and right coronary artery (RCA). There were significant differences in the distribution of IRA and the numbers of vascular lesions between the two groups (*P* < 0.05). Specifically, the proportion of ATRBBB group to have LAD as IRA was higher (90.0%). The TRBBB group was more likely to have RCA as an IRA (76%). In the TRBBB group, single vascular lesions were dominant (72.1%), while in the ATRBBB group, vascular lesions were more evenly distributed. In addition, there was no significant difference in the IRA anterior TIMI0/1, occlusion (proximal or nonproximal), and the proportion of stent implantation in emergency PCI between the two groups. Figure 1 shows coronary angiography graphs of two representative AMI cases combined with new-onset TRBBB and new-onset ATRBBB.

### 3.4. Clinical Outcomes

#### 3.4.1. In-Hospital MACE

Among the 224 patients in this study, 93 cases of MACE occurred in hospital, including 21 cases in the TRBBB group and 72 cases in the ATRBBB group [OR = 5.929, 95% CI (3.247–10.826), *P* < 0.001] (Table 4). ATRBBB group has a higher ratio of cardiac shock, malignant ventricular arrhythmia, and sudden cardiac death. On the other hand, TRBBB group has a higher ratio of type II and above serious AVB.

Univariate logistic regression was used to screen out the predictors of in-hospital MACE in AMI patients combined with new-onset RBBB, including age, sex, BMI, alcohol, hypertension, diabetes, hyperlipemia, OMI, Killip ≥ II, CK-MB peak, LVEF%, TIT, ATRBBB, STEMI, transient RBBB, anterior/anterior septum/extensive anterior wall, LAD as IRA, the number of vascular lesions, and PCI. The result showed that age, ATRBB, transient RBBB, TIT, OMI, Killip ≥ II, CK-MB peak, LAD as IRA, the number of vascular lesions, and PCI had significance for predicting in-hospital MACE. The above results were further analyzed by the multifactor logistics stepwise regression, and the results showed that the ATRBBB, TIT, 3-vessel lesion, OMI, and Killip ≥ II were independent predictors of in-hospital MACE in patients with AMI combined with new-onset RBBB (Table 5).

#### 3.4.2. One-Year Survival Analysis

During the follow-up of 365 days (one year), there were 48 (22.4%) cases of death: 4 (3.8%) cases in TRBBB group and 44 (36.7%) cases in ATRBBB group. There was an obvious difference between the two groups as regards the 1-year mortality rate [HR: 11.577 (95% CI 4.157–32.24),*P* < 0.001]. The 1-year K-M curve is shown in Figure 2. Cox survival analysis was used to screen independent predictors of 1-year survival in patients with AMI complicated with new-onset RBBB, and the results showed that age, ATRBB, ITI, and three-vessel lesion are independent predictors of 1-year survival of AMI patients combined with new-onset RBBB (Table 6).

## 4. Discussion

AMI is an acute and severe disease that threatens humans' health [14, 15]. The principle of AMI treatment is to open IRA early, completely, and continuously to reduce the scope of myocardial necrosis to reduce its mortality and improve its prognosis [8]. Therefore, early diagnosis of AMI is particularly important for emergency treatment. ECG has a special value in early diagnosis, warning, and prognosis of AMI. Main previous AMI guidelines indicated that the dynamic changes of ST-T and the new-onset LBBB should be indications for early emergency revascularization of AMI [6, 7]. In recent years, many clinical studies have proposed that AMI patients combined with BBB have a poor prognosis, and the incidence of AMI combined with new-onset RBBB is higher than LBBB [10, 16]. The emergence of new-onset RBBB can also mask ST elevation, such as when LBBB affects the early diagnosis of AMI [17, 18]. Therefore, the value of new RBBB in the early stage of AMI diagnosis has received extensive attention. Finally, in the 2017 ESC guidelines of STEMI, new-onset RBBB was considered as an indication of emergency revascularization together with new-onset ST-segment elevation and LBBB [8]. As early as 2010, our team proposed the importance of new-onset RBBB in AMI and suggested that it is an indication for emergency revascularization [9]. Based on years of clinical summary, we found that patients with AMI combined with RBBB showed differences in graphics. Some patients showed typical graphics in accordance with the diagnostic criteria of RBBB, whereas others showed atypical graphics that did not fully accord with the diagnostic criteria of type RBBB, such as R wave or qR type on the V_1_/V_2_ lead. The coronary artery lesion characteristics and clinical prognosis of patients with two kinds of RBBB patterns seemed to be different. Therefore, this study included AMI patients with new-onset RBBB in our team in the past 10 years. We divided them into TRBBB and ATRBBB groups according to their RBBB ECG graphic characteristics. The clinical baseline, coronary artery lesion characteristics, and prognosis of patients in the two groups were compared to determine the differences in emergency revascularization and prognosis between the two groups.

The proportion of all RBBB in patients with AMI was 9.7%, and new-onset RBBB was 8.43%, slightly higher than those in previous studies [4, 7]. The proportion of ATRBBB in patients with AMI combined with RBBB was 53.57%. The pattern of BBB on ECG is caused by the asynchronous conduction between left and right ventricles. Theoretically, it is believed that if the conduction difference between the left and right ventricles is more than 40 ms, the ECG will manifest a BBB graph. The conduction obstacle may occur in the left or right bundle branches, Purkinje fibers, or myocardium. In terms of branch anatomy [19], the right branch mainly runs in the front 1/3 of the interventricular septum; its main blood supply comes from the anterior descending branch. The left branch also runs in the interventricular septum, but the blood supply of the left branch origins from the anterior descending and posterior descending branches; it has a double blood supply. When AMI occurs, the incidence of RBBB is actually higher than that of LBBB. On the other hand, if the blood supply of the left ventricle or the right ventricle muscle drops sharply in a short period of time, the conduction of electrical activity between the two ventricles will be different, resulting in the BBB graph in ECG due to the difference of intramuscular electrical conduction between the left and right ventricles rather than left or right branch bundles run in the ventricular septum. Therefore, AMI combined with new-onset RBBB may be caused by LAD occlusion affecting the blood supply of the right fasciculus branch which runs through the septum or RCA proximal occlusion affecting the blood supply of right ventricular blood branch originating from RCA, affecting Purkinje fiber depolarization and intracellular depolarization of right ventricular subendocardium, resulting in delayed right ventricular contraction. From anatomical and electrophysiological mechanism aspects, the abnormal function of the real right bundle branch is due to the LAD proximal occlusion leading to its blood supply affection, but the conduction delays in the right Purkinje fibers or myocardium is due to right ventricle blood supply affected. Both reasons above can lead to new-onset RBBB graph in the ECG. This study only distinguished TRBBB and ATRBBB from EGG graphics performance, not perfectly matching the anatomical and electrophysiological mechanism. In conclusion, the proximal occlusion of LAD or RCA can lead to new-onset RBBB in the ECG but with a different mechanism.

The results of this study showed that TRBBB is 53.57% in AMI combined with new-onset RBBB, and ATRBBB is 46.43%. Compared with TRBBB, ATRBBB has a higher proportion of anterior/anterior septum/extensive anterior wall infarction (IRA is LAD). The main difference between TRBBB and ATRBBB on the ECG is that the initial depolarizing wave disappears in the initial 40 ms of QRS wave, instead of q or Q wave, and qR or QR pattern appears. The reason for the above phenomenon is the occlusion of the LAD proximal segment, which affects the blood supply of the anterior septal branch originating from LAD, resulting in ischemic necrosis or transient function losing of the right bundle branch running in the anterior ventricular septum. If the ischemic time is long enough, the interventricular septum necrosis leads to the formation of pathological Q waves in the first 40 ms in V_1_/V_2_ leads. Thus, the typical RBBB pattern of rsR′ will evolve into an qR or QR pattern named ATRBBB in this research due to the long ischemic time of the interventricular septum. If the total occluded time LAD is short and pathological Q wave in V_1_/V_2_ leads cannot be formed, TRBBB will present, which is consistent with the shorter total ischemic time in the TRBBB group than in the ATRBBB group in this research. The reason above can explain why 22.4% of patients with proximal occlusion LAD presented typical RBBB in this study, and 53.13% of these typical RBBB combined with LAD occlusion presented transiently, which was related to the reversible injury of the right bundle branch due to short ischemic period.

RCA proximal occlusion affects the blood supply of the right ventricle and the inferior wall of the heart; thus pathological Q waves mostly present in the inferior wall and right ventricle leads to ECG. The occurrence of transient RBBB may be due to the late depolarization of the right ventricle compared with the left ventricle. Therefore, there are anatomical and electrophysiological mechanisms differences between anterior wall myocardial infarction with permanent ATRBBB and the inferior wall myocardial infarction with transient TRBBB. Other scholars proposed that obstruction of proximal RCA blood flow leading to right ventricular dilation, mechanical stretching, and possible preexisting chronic injury of the right bundle branch are other causes of new-onset RBBB in inferior myocardial infarction [20].

The results of this study suggested that some patients in both the TRBBB group and the ATRBBB group have not shown typical dynamic ST-segment elevation. Although there was no statistically significant difference in the proportion of dynamic ST-segment elevation between the two groups, the proportion of ST-segment elevation in the TRBBB group was higher than that in the ATRBBB group. This may be related to the higher proportion of IRA was RCA in the TRBBB group. Proximal RCA occlusion led to ST-segment elevation in the inferior wall leads, and changes in secondary repolarization in RBBB mostly affect ST-T of anterior/anterior septum wall leads. Therefore, the false normalization of ST-T of the anterior/anterior septum wall leads to myocardial infarction combined with RBBB may mask ST-segment elevation and the early stage of AMI, affecting the early diagnosis. Some authors warn that minor ST elevations in the anterior leads (V_1_–V_4_) can be missed due to compensation by pseudonormalization of the negative T waves [21]. Widimsky et al. showed that, even in large infarcts (caused by left main or proximal LAD coronary artery occlusion), bifascicular block (RBBB + LAH or rarely RBBB + LPH) may occur without typical STE [22]. Therefore, we should not request ST-segment elevations to be present for the diagnosis of AIM with RBBB to initiate emergency revascularization.

Compared with the TRBBB group, the ATRBBB group had a higher proportion of worse cardiac function, a higher peak value of CK-MB, lower LVEF%, longer TIT, and a higher proportion of multivessel lesions. AMI combined with new-onset ATRBBB means larger infarction scope and worse heart function than the TRBBB group. In addition, compared with the TRBBB group, the ATRBBB group had a higher proportion of in-hospital MACE and 1-year all-cause mortality. ATRBB group had a higher proportion of cardiac shock and malignant arrhythmia in the hospital, which may be associated with larger infarction scope. The higher proportion of type II and above serious AVB in the TRBBB group is due to the blood supply of atrioventricular nodes originating from RCA mostly. TRBBB group had a higher proportion of RCA as IRA. Multivariate logistic regression and multivariate COX survival analysis of in-hospital MACE and 1-year death showed that ATRBBB was an independent predictor of in-hospital MACE and 1-year death in AMI patients combined with new-onset RBBB. As the results mentioned above, AMI patients with new-onset ATRBBB in ECG have a worse clinical prognosis compared to those in the TRBBB group.

## 5. Conclusion

In summary, compared with the TRBBB group, patients in the ATRBBB group had poorer prognosis both in hospital and within 1 year. New-onset ATRBBB was an independent predictor of in-hospital MACE and 1-year death in patients with AMI combined with RBBB. The anterior wall myocardial infarction combined new typical RBBB hints ischemia with early stage, regardless of whether there was ST-segment elevation or not, and timely revascularization should be activated to reduce myocardial injury, retain the right bundle branch function, reduce the infarction area, and improve clinical prognosis.

## Figures and Tables

**Figure 1:** Two representative cases of AMI combined with new-onset TRBBB and ATRBBB. (a) One inferior wall AMI case presented TRBBB in the ECG (red arrow pointed rsR′ graph in lead V_1_). (b) Emergency CAG showed total occlusion in the proximal segment of RCA (red arrow marked occlusion site). ((c) and (d)) The RCA was opened after primary PCI (red arrow showed distal blood flow was restored). (e) One anterior and anterior septum wall AMI case presented ATRBBB in ECG (red arrow pointed qR′ graph in lead V_1_). (f) Emergency CAG showed total occlusion in the proximal segment of LAD (occlusion site was marked by a red arrow). (g) The LAD was opened after primary PCI (red arrow showed distal blood flow was restored).

**Figure 2:** K-M curve of 1-year survival analysis in the two groups.

**Table 1:** Clinical characteristics at baseline.

Variable	TRBBB group (*n* = 104)	ATRBBB group (*n* = 120)	*P* value
Ages (*Y*)	65.63 ± 11.72	65.73 ± 12.60	0.50
Males (*n*/%)	67.3	77.5	0.087
BMI (kg/m^2^)	27.76 ± 2.59	28.67 ± 2.79	0.013^*∗*^
Smoking (%)	56.7	69.7	0.044^*∗*^
Alcohol (%)	51.9	65.8	0.035^*∗*^
Hypertension (%)	60.6	66.7	0.344
Diabetes (%)	38.5	50.8	0.063
Hyperlipemia (%)	91.3	90.8	0.893
OMI (%)	16.3	203.3	0.193
Killip ≥ II (%)	16.3	42.5	<0.001^*∗*^
CK-MB peak (U/L)	245.82 ± 93.66	347.55 ± 118.87	<0.001^*∗*^
LVEF (%)	48.39 ± 6.34	44.19 ± 6.75	<0.001^*∗*^
TIT (h)	6.91 ± 3.47	10.78 ± 4.60	<0.001^*∗*^

Values are given in % or mean ± standard deviation. BMI, body mass index; EF, ejection fraction; OMI, old myocardial infarction; TIT, total ischemic time. ^*∗*^Statistical value.

**Table 2:** ECG characteristic differences between TRBBB and ATRBBB group.

Value	TRBBB group (*n* = 104)	ATRBBB group (*n* = 120)	*P* value
STEMI (%)	81.7	72.5	0.103
Transient RBBB (%)	65.4	5.8	<0.001^*∗*^
Anterior/anterior septum/extensive anterior wall (%)	24.0	90.0	<0.001^*∗*^

Values are given in %. STEMI: ST-segment elevation myocardial infarction. ^*∗*^Statistical value.

**Table 3:** Coronary artery characteristics and PCI difference between TRBBB and ATRBBB groups.

Values	TRBBB group (*n* = 104)	ATRBBB group (*n* = 120)	*P* value
IRA (%)			<0.001^*∗*^
LM	0	0	
LAD	24.0	90	
RCA	76.0	10	
LCX	0	0	
Numbers of vascular lesions (%)			<0.001^*∗*^
1-vessel	72.1	35.0	
2-vessel	13.5	36.7	
3-vessel	14.4	28.3	
IRA proximal occlusion (%)	98.1	97.5	0.388
IRA anterior TIMI0/1 (%)	84.6	80.0	0.245
Emergency PCI	92.4	90.0	0.245

Values are given in %. IRA: infraction related artery; LM: left coronary artery; LAD: left anterior descending coronary artery; RCA: right coronary artery; LCX: left circumflex coronary artery; TIMI: thrombolysis in myocardial infarction; PCI: percutaneous coronary intervention. ^*∗*^Statistical value.

**Table 4:** In-hospital MACE difference between TRBBB and ATRBBB groups.

Values	TRBBB group (*n* = 104)	ATRBBB group (*n* = 120)	*P* value
In-hospital MACE (%)	20.2 (21)	60 (72)	<0.001^*∗*^
Cardiac shock	3.8	25.9	<0.001^*∗*^
Malignant ventricular arrhythmia	3.8	15.8	0.03^*∗*^
Type II and above serious AVB	8.7	2.5	0.043^*∗*^
In-hospital recurrent AMI	1.9	5.0	0.29
Sudden cardiac death	1.9	10.8	0.008^*∗*^

Values are given in %. MACE, major advent cardiac event. AVB, atrial ventricular block. ^*∗*^Statistical value. AMI, acute myocardial infarction.

**Table 5:** Multifactor logistic regression of independent predictors of in-hospital MACE in AMI patients combined with new-onset RBBB.

Values	*P* value	OR (95% CI)
ATRBBB	0.048^*∗*^	3.634 (1.011–13.068)
Age	0.112	1.030 (0.993–1.068)
Transient RBBB	0.661	0.742 (0.195–2.818)
CK-MB peak level	0.704	1.001 (0.996–1.006)
LAD as IRA	0.988	0.99 (0.252–3.884)
3-vessel lesion	0.042^*∗*^	3.137 (1.044–9.427)
TIT	0.001^*∗*^	1.323 (1.115–1.569)
OMI	0.031^*∗*^	3.569 (1.124–11.335)
Killip ≥ II	0.005^*∗*^	4.702 (1.612–13.718)
PCI	0.234	0.406 (0.092–1.791)

LAD, left anterior descending branch. IRA, infarction related artery. TIT, total ischemia time. OMI, old myocardial infarction. PCI, percutaneous coronary intervention.

**Table 6:** Cox analysis independent predictors of 1-year mortality in AMI patients combined with new-onset RBBB.

Value	*P* value	HR (95% CI)
Age	0.009^*∗*^	1.046 (1.011–1.083)
Transient RBBB	0.918	1.092 (0.207–5.768)
ATRBBB	0.041^*∗*^	6.718 (1.084–41.635)
TIT	0.004^*∗*^	1.119 (1.037–1.207)
OMI	0.933	0.937 (0.506–1.807)
Killip ≥ II	0.138	1.969 (0.804–4.820)
CK-MB peak level	0.256	1.002 (0.998–1.006)
LAD as IRA	0.389	0.492 (0.098–2.467)
3-vessel lesion	0.026^*∗*^	4.433 (1.192–16.492)

LAD, left anterior descending branch. IRA, infarction related artery. TIT, total ischemia time. OMI, old myocardial infarction. PCI, percutaneous coronary intervention.

## Data Availability

The data used to support the findings of this study are available from the corresponding author upon request.
